The article "The Effect of Routine Management Combined with Case Management Model on Social Support, Self-Efficacy, Self-Management Ability, and Psychological Flexibility of AIDS Patients" was retracted in 2023. Reasons: unreliable results or conclusions; lack of ethics approval or compliance; concerns about the data; concerns about the peer review.

# The Effect of Routine Management Combined with Case Management Model on Social Support, Self-Efficacy, Self-Management Ability, and Psychological Flexibility of AIDS Patients

**DOI:** 10.1155/2022/9213877

**Published:** 2022-08-04

**Authors:** Li Liu, Jing Zhou, Huan Xiao, Yanhe Luo, Yan Zeng, Li Fan, Chen Zheng

**Affiliations:** ^1^Department of Infectious Diseases, Jinyintan Hospital, Wuhan, China 430000; ^2^Department of Dermatology, Huangshi Central Hospital, Affiliated Hospital of Hubei Polytechnic University, Edong Healthcare Group, Hubei Key Laboratory of Kidney Disease Pathogenesis and Intervention, China

## Abstract

**Objective:**

To explore the influence of conventional management combined with case management on social support and self-efficacy of AIDS patients.

**Methods:**

The clinical case data of 120 AIDS patients who were treated and nursed in our hospital from June 2019 to June 2021 were selected as the research objects and were divided into the control group and the observation group according to the digital table method, with 60 cases each. The control group implements routine management, and the observation group implements case-based nursing management on this basis and compares the effects of self-efficacy, self-management ability, nursing ability, social support, and psychological flexibility of the two groups of patients.

**Results:**

Before the intervention, the quality of life scores of the two groups was not statistically significant (*P* > 0.05). After the intervention, the physical function score, pain management score, and symptom response score of the observation group were significantly higher than those of the control group, and statistics showed that the difference was statistically significant (*P* < 0.05). Before the intervention, the self-management ability of the two groups of patients was not statistically significant (*P* > 0.05). After the intervention, the observation group's symptom management, emotional cognition management, social support and assistance, daily life management, disease knowledge management, and treatment compliance management were significantly higher than those of the control group. Statistics show that this difference is statistically significant (*P* < 0.05). Before the intervention, there was no significant difference in the nursing ability and psychological flexibility between the two groups of patients (*P* > 0.05). After the intervention, the observation group's health knowledge level, self-care skills, self-care responsibility, self-concept, and mental flexibility (resilience, strength, optimism) indicators were higher than the control group, while the depression mood disorder score was significantly lower than the control group; statistics showed that this difference was statistically significant (*P* < 0.05).

**Conclusion:**

Routine management combined with case-based nursing management can effectively improve the self-management ability and psychological flexibility of AIDS patients, improve patient care ability and self-efficacy, and provide certain reference value for effective management of AIDS patients.

## 1. Introduction

AIDS is a chronic infectious disease caused by the human immunodeficiency virus. Studies have shown that since the first case of AIDS patients was discovered in the United States, AIDS has spread rapidly around the world, and the current epidemic trend of AIDS has long become a key issue of global concern [1]. The main routes of AIDS transmission are intravenous drug transmission and sexual transmission. The AIDS epidemic in the whole region is generally stable, but the prevention and control situation is still severe. The concept of case management was first proposed in the 1970s and first introduced in the United States [2]. The American Case Management Association defines the process of case management as a cooperative treatment and medical service procedure including evaluation, planning, implementation, coordination, supervision, and evaluation. Mainly through communication and coordination with patients, medical institutions make full use of effective resources to meet the health needs of patients and ultimately achieve the purpose of providing patients with high-quality medical services and reasonable fees [3]. Case management is a nursing model produced in the implementation of the biopsychosocial medicine model and the medical resource control management system. It meets the needs of clinical, community, and market [4]. Compared with the conventional management mode, case management is patient-centered, and the medical institution and the patient jointly manage the disease. It has the characteristics of humanization, individualization, and strong pertinence [5]. By constantly understanding the actual needs of patients and their families, working with patients to formulate personalized medical service plans, real-time tracking, and monitoring of patients' treatment conditions will help to achieve overall and continuous care for patients and can effectively compensate insufficiency of the conventional management model [6]. In addition, compared with other diseases, AIDS patients and AIDS itself have certain specificities and sensitivities. The patient's condition and behavior are directly related to the development of their lives, families, and even society. The implementation of effective management strategies for AIDS patients is of far-reaching significance [7]. Therefore, this study explores the impact of conventional management combined with case management on the social support, self-efficacy, self-management ability, and psychological flexibility of AIDS patients and provides a reference for the management of AIDS patients.

## 2. Information and Methods

### 2.1. Research Object

The clinical case data of 120 AIDS patients who were treated and nursed in our hospital from June 2019 to June 2021 were selected as the research objects, and the patients who met the inclusion criteria were numbered according to the order of care, and the third edition was used. The screening process for included patients is shown in Figure 1. The number table method of “Medical Statistics” [8] was randomized into a control group and an observation group with 60 cases each. In the observation group, there were 28 males and 32 females, aged 25-63 (39.93 ± 10.19) years old, body mass index 19.2-28.5 (23.32 ± 2.59) kg/m^2^. In the control group, there were 20 males and 40 females, aged 21-61 (36.48 ± 9.37) years old, body mass index 19.0-28.7 (23.33 ± 2.51) kg/m^2^. There was no statistically significant difference in baseline information between the two groups (*P* > 0.05), and they were comparable.

### 2.2. Exclusion Criteria

Inclusion criteria are as follows: (1) the selected patients meet the diagnostic criteria of the “Expert Consensus on the Diagnosis and Treatment of Human Immunodeficiency Virus/AIDS Patients with Nontuberculous Mycobacterial Infection” [9], and the AIDS patients have clear consciousness and can speak normally; (2) HIV antibody confirmation test is positive or HIV strain is isolated from the blood, with acute HIV infection syndrome or epidemiological history, and two HIV nucleic acid test results at different times are both positive; (3) and HIV infection and CD4 + T Lymphocytes 200/mm^3^, HIV infection, and at least one adult AIDS-indicative disease. Exclusion criteria are as follows: (1) those who suffer from malignant tumors are in critical condition or are accompanied by severe complications, are detained in violation of the law, have severe cognitive dysfunction, and cannot cooperate; (2) those who have severe complications, those with mental disorders, and those with communication disorders; and (3) patients with severe trauma, such as severe head injury and thoracolumbar fracture, history of drug allergy, and history of major surgery.

### 2.3. Method

#### 2.3.1. Routine Management

The control group implements routine management, that is, the establishment of health files including general information such as the patient's name, gender, ethnicity, and marital status. The doctor in charge will follow up the patients via telephone or face-to-face communication, each time for 5-10 minutes. The content includes informing the patient of the results of the latest examination and the time of the next follow-up, asking about the patient's body weight, medication compliance, and whether there are complications, etc., providing the patient with basic knowledge of drugs, and improving bad behaviors (such as drug use and multiple sexual partners). Psychological management: (1) listening: the most important and basic step in psychological counseling is to listen. Nurses take observational interviews, interviewing AIDS patients on topics such as the cause, course, work, social interaction, and life patterns of AIDS patients. Pay attention to the conversation. When it comes to privacy, the nurse should respect the patient and should not show expressions of surprise or surprise; if the patient is emotional and it is not conducive to continuing the conversation, the nurse can change the topic in time or guide the patient's negative emotions. (2) Thinking: in-depth listening helps nurses understand the patient's mental state and self-expectations, judge the patient's needs for disease, empathize in the follow-up interviews, analyze the reasons for the patient's different mental states such as loneliness, depression, and anger, and actively help the patient to educate the patient negative emotions. (3) Expression: after collecting the patient's negative emotions and analyzing the causes, nurses should rationally express their concern for the patient. On the one hand, they should resonate with the patient's negative emotions, allowing the patient to feel their sincere concern and prompting the patient to accept the nurse. And take the initiative to cooperate with the nurse's treatment; on the other hand, if the patient and his family have unreasonable behavior or request, the nurse should rationally refuse to accept and can not blindly cater to the needs of the patient. In addition, nurses also need to express their extreme emotions rationally. Regarding self-denial, self-doubt, sensitive and suspicious, etc., nurses should correctly encourage patients to express their needs and at the same time guide patients to reflect on themselves so that patients can think and express correctly. Transform passive thinking and passive acceptance into active thinking, active understanding, and initiative to propose ideas.

#### 2.3.2. Case Nursing Management

The observation team implements case care management on this basis, namely, (1) preparation: set up a case care management team: 1 case manager, 3 AIDS specialists, 1 psychological counselor, 1 nutritionist, and 1 pharmacist. It is composed of 1 professional nurse, 2 volunteers; 4 Han nationality, 3 Uygur nationality, 1 Hui nationality, and 2 Kazakh nationality. The main work content of the case care management team: the case manager is responsible for assessing patients' health problems, formulating management plans, determining management issues, monitoring the completion of management measures, coordinating the work assignments of members of the team, etc.; medical experts in the AIDS field are responsible for formulating patient treatment plans and complete outpatient and telephone follow-up of patients; specialist nurses are responsible for establishing case management files, which include patient's name, gender, age, treatment number and other general information, patient follow-up schedule, case management process sheet, and various examination records. Volunteers are responsible for contacting and organizing peer education activities. All members in the group are required to be familiar with the case management process and operation methods and to clarify their own work content. Minority patients are designated to be responsible for the team members of the same ethnic group who can communicate smoothly with them. Psychological counselors are responsible for guiding the patients and their families' unhealthy psychological problems. The teacher is responsible for drug management; the nutritionist is responsible for dietary adjustments for patients with underweight and poor nutritional status.

Specific implementation: (1) evaluation: before the patient starts antiviral treatment, during the outpatient follow-up, the management team members will adopt face-to-face communication to collect and evaluate the patient's information, including basic information of the patient, current disease status, self-management ability, and psychology elasticity level. (2) Formulation of a case management plan: the management team discusses the issues that the patient needs to manage based on the evaluation results, and the case manager integrates the opinions of the team to formulate a case management plan with the patient, including daily life management, behavior standard management, disease knowledge management, problems in symptom management, treatment compliance management, and emotional cognitive management. (3) Take intervention measures: inform patients to follow up in outpatient clinics on time at 1 month, 2 months, 3 months, and 6 months after the start of antiviral therapy. Each follow-up time is 30-50 minutes. Specialists will use face-to-face interviews to evaluate the treatment effect and improve the treatment plan. Specialized nurses distribute bilingual educational materials with pictures and texts to patients and combine the materials to carry out health education on self-management-related knowledge, such as basic knowledge of AIDS, the importance of medication compliance, and the correct use of condoms. When patients have psychological problems such as pessimism, depression, and fear, specialist nurses and psychologists will jointly provide psychological counseling to them to enhance the patients' confidence and ability to resist the disease and stimulate the patients' self-care awareness. The specialists will conduct regular telephone follow-ups with the patients, including the completion of the follow-up time and reminders of the abnormal results of the latest examination, understanding the patient's recent physical condition, medication compliance, and whether there are other needs, etc., and make detailed records. Follow-up frequency: the patient will be followed up once a week in the first month of starting medication; in the second and third months, once every two weeks; in the fourth, fifth, and sixth months, every month follow up 1 time. The case manager establishes a WeChat group to regularly send self-management-related knowledge information to patients at a frequency of twice a week until the patient has been managed for 6 months. During this period, if the patient has any questions, the team members will give answers in time. If the patient is unable to use WeChat, record the WeChat account of their trusted family members or friends, and require that health knowledge be communicated to the patient in a timely manner. If the patient has difficulty typing, he can communicate by voice. Inform patients that they need to respond in time after receiving the WeChat education content. If the patient does not reply to the message within 1 week, the case manager will conduct a telephone return visit to ensure the patient's participation. For patients with poor compliance, volunteers are responsible for carrying out peer education activities, choosing patients who are similar to their family backgrounds and disease conditions, actively cooperate with treatment, have good treatment effects, and volunteer to participate in voluntary activities. Difficult patients build confidence in treating diseases and improve treatment compliance and self-management capabilities.

### 2.4. Observation Indicators

(1) Self-efficacy: the self-efficacy scale (CPSS) was used to evaluate the self-efficacy of the two groups of hemodialysis patients after intervention. The content mainly includes physical function, pain management, and symptom response. The higher the score of the patient, the stronger the self-efficacy. The internal consistency reliability coefficient of the scale is 0.896, the Guttmann split-half reliability is 0.763~0.896, and the test-retest reliability is 0.810~0.902. (2) Self-management scale contains 49 items, including daily life management (8 items), life behavior standards (6 items), disease knowledge management (4 items), symptom management (9 items), treatment compliance management (8 items and 7 items), emotional cognitive management (6 items), and seeking social support and help (8 items). Using the Likert 5-level scoring method, “no” is counted as 1 point, “rarely” is counted as 2 points, “sometimes” is counted as 3 points, “often” is counted as 4 points, and “always” is counted as 5 points. The total score ranges from 49 to 245 points. The higher the score, the higher the patient's self-management ability. The content validity of the scale is 0.939, and the content consistency coefficient Cronbach's *α* coefficient is 0.8535. The Cronbach's coefficient of the scale in this study was 0.872. (3) Self-care ability assessment form includes 46 items in 3 dimensions, namely, health knowledge level (14 items), self-care skills (12 items), and self-care responsibility (8 items). Each item has 5 points, 11 of which are reverse scores, with a full score of 172 points. The higher the score, the stronger the self-care ability. (4) Psychological resilience: there are 25 items in the psychological resilience scale, including three factors: resilience (13 items), strength (8 items), and optimism (4 items). The Likert 5-level score is used, and 0 ~ 4 points are assigned from “never” to “almost always,” respectively. The score ranges from 0 to 100 points; the higher the score of the description, the better the psychological flexibility. The scale has been used in outpatients, mental disorders, cancer patients, etc. The internal consistency reliability Cronbach's *α* coefficient is 0.91, and the Cronbach's *α* coefficient of each factor is 0.60~0.888. The patient fills in independently without being affected by any internal or external factors, and the test will be completed within 60 minutes.

### 2.5. Statistical Methods

Use EpiData to enter all the data, and then, use SPSS 25.0 to statistically process the data. The data needs to be entered into a computer database by a second person to ensure the completeness and accuracy of the data. The measurement data represented by the mean ± standard deviation$\bar{x}\pm s$ using the one-way variance test and the counting data represented by the percentage (%) using the *χ*^2^ test are statistically significant at *P* < 0.05.

## 3. Results

### 3.1. Comparison of Self-Efficacy

Before the intervention, the comparison of the quality of life scores of the two groups of patients was not statistically significant (*P* > 0.05). After the intervention, the physical function score, pain management score, and symptom response score of the observation group were significantly higher than those of the control group, and statistics showed that the difference was statistically significant (*P* < 0.05) (see Table 1).

### 3.2. Comparison of Self-Management Capabilities

Before the intervention, the self-management ability of the two groups of patients was not statistically significant (*P* > 0.05). After the intervention, the observation group's symptom management, emotional cognition management, social support and assistance, daily life management, disease knowledge management, and treatment compliance management were significantly higher than those of the control group. Statistics show that this difference is statistically significant (*P* < 0.05) (see Table 2).

### 3.3. Comparison of Nursing Ability and Psychological Flexibility

Before the intervention, there was no significant difference in the nursing ability and mental flexibility between the two groups of patients (*P* > 0.05). After the intervention, the observation group's health knowledge level, self-care skills, self-care responsibility, self-concept, and mental flexibility (resilience, strength, optimism) indicators were higher than the control group, while the depression mood disorder score was significantly lower than the control group; statistics showed that this difference was statistically significant (*P* < 0.05) (see Tables 3 and 4).

## 4. Discussion

After the intervention of this study, the physical function scores, pain management scores, and symptom response scores of the observation group were significantly higher than those of the control group, indicating that routine management combined with case care management can effectively improve the self-efficacy of AIDS patients. Due to the particularity of the transmission method of AIDS and the infected population, AIDS patients not only have to endure the pain caused by the disease itself but also worry that they may become the source of infection for the surrounding population [10]. It is easy to produce negative emotions in its psychology and behavior, which in turn causes the patient's sense of self-efficacy to decline and cannot cope with existing health problems [11]. Studies have shown that by enhancing patients' self-efficacy, AIDS patients can be motivated to cooperate with treatment and care, and their confidence and ability to fight disease can be stimulated to stimulate patients' self-care awareness [12]. In this study, while the case team members educate the patients on self-management, they also communicate with the patients, and the number of exchanges has increased, and they have been patient and meticulous psychological counseling [13]. In addition, according to the wishes of the patients, peer education was adopted to organize the watching of positive and positive case videos and volunteers to speak out and conduct psychological consultations, etc., to continuously guide patients to reduce their own pressure and enable patients to find the meaning and value of self-existence, so as to actively cooperate with treatment and manage their own health problems [14].

After the intervention of this study, the observation group's symptoms management, emotional cognitive management, social support and assistance, daily life management, disease knowledge management, and treatment compliance management were significantly higher than those of the control group, indicating that routine management combined with case care management can effectively improve AIDS. The reason for the analysis may be that only the investigation of infectious disease hospitals was carried out, and the sample has limitations. Xinjiang is a multiethnic area, and there are some differences in population distribution, customs, and language environments among different ethnic groups [15]. Compared with the conventional hospital management model, the case management model can combine the essentials of AIDS prevention and control work to provide patients with more personalized management services and professional support, which has the characteristics of strong individualization and strong pertinence [16]. In addition, this model plays a very important role in promoting effective self-health management of patients, improving patient compliance and quality of life, strengthening the cooperation of medical-related teams, and improving their work efficiency [17]. There may be insufficient communication between medical staff and patients, and patients lack understanding and acceptance of the self-management content mastered by patients, which can be seen from the two dimensions of the low score rate [18]. AIDS patients tend to neglect daily life management including diet, smoking, drinking, sleep, and exercise. In addition, there is obvious discrimination against AIDS-infected people in society. Most patients are unwilling to let others around after they become ill. After knowing their condition, they are reluctant to ask for help from others, so they cannot get help from others [19]. Therefore, it is recommended that medical staff should take the patient as the center and provide personalized health guidance and assistance, such as designating medical staff of the same ethnicity or gender as the patient to conduct self-management education on medication compliance, symptom management, life behavior, etc., in order to continuously improve patients' awareness of the disease [20]. At the same time, provide patients with adequate medical information and emotional support. In the case of the patient's informed consent, the patient can communicate with the person voluntarily informed to help the patient establish a good social support system, promote the patient's awareness of self-management, and improve the self-management ability [21]. In this study, the case management team is patient-centered, and through evaluation and discussion of the patient's family status, disease status, self-management ability, etc., the case manager and the patient jointly formulate a management plan. The members of the case management team provided patients with bilingual publicity materials for health education and used WeChat counseling, telephone follow-up, peer education, and organization of volunteer activities to provide personalized health guidance and assistance to patients. At the same time, they took AIDS specialists. Subsequently, multidisciplinary approaches such as pharmacy, psychology and nutrition are used for treatment [22]. Enable medical staff to communicate with patients and their families in depth; constantly understand the needs of patients and do their best to provide patients with support including medical care, economics, interpersonal relations, and information; and effectively improve patients' self-management capabilities [23].

After the intervention of this study, the observation group's health knowledge level, self-care skills, self-care responsibility, self-concept, and mental flexibility (toughness, strength, optimism) indicators were higher than those of the control group, while the depression mood disorder score was significantly lower than that of the control group, indicating that the routine management and case-based nursing management can effectively improve the psychological flexibility of AIDS patients and improve the patient's nursing ability. Good psychological flexibility can effectively reduce the negative impact of the disease itself and external factors on the patients and can significantly reduce the patients' psychological stress response and promote the patients to adapt to the status quo faster and better. AIDS patients need to take medicine for life and cannot be cured, and there is a certain particularity in the mode of transmission [24]. Therefore, AIDS patients tend to have bad feelings such as inferiority, fear, and pessimism in their psychology and behavior. Studies have shown that positive personality traits, family and social support, and the provision of external resources are protective factors that enhance the psychological resilience of patients [25]. By changing the cognitive level of patients, they can relieve painful emotions, return to normal life from the shadows as soon as possible, and better adapt to and accept the current situation. At the same time, psychological resilience is also the main factor that affects the self-management ability of AIDS patients, and there is a close positive correlation between the two; that is, the higher the psychological resilience level, the more effective the patients can cope with the negative impact of the disease and actively cooperate with the treatment and take measures that are conducive to the recovery of the disease. [26]. This reminds medical staff that when following up patients, in addition to repeatedly emphasizing the importance of medication compliance and improving bad lifestyles, they also need to inform patients that the development of the disease is controllable based on the medication prescribed by the doctor, to establish the confidence of patients in active treatment [27–29]. At the same time, patients should be encouraged to return to society and participate in more social activities to build a patient's psychological elastic support system and enhance the patient's ability to adapt. Through communication and exchanges with patients, the members of the case management team constantly understand the psychological needs of patients and implement targeted intervention strategies [30–33]. The case manager will arrange the patient for psychological consultation in time to relieve the pessimism and make the patient feel respected, valued, and understood. At the same time, in compliance with the patient's wishes, communicate with their family members and trusted personnel to help the patient obtain the understanding of those around him, continuously stimulate the patient's psychological flexibility by mobilizing external forces such as family and society, and enhance the patient's ability to adapt to the current situation, so as to encourage them to maintain an optimistic attitude and actively cooperate with treatment [34, 35].

This research is innovative and has some limitations. This study uses a randomized controlled trial. In the intervention of the two groups of subjects, there may be confounding factors, which may cause bias. Therefore, in future research work, try to control various interference factors to make the research results more real and reliable. The implementation of the case management model should be a long-term persistent management method. However, due to time constraints, the intervention period for patients in this study is relatively short. It is hoped that this model can be implemented for a long time in the future, and the intervention time can be extended to explore the advantages of the case management model and improve the effectiveness of self-management ability and quality of life of AIDS patients. It is recommended to repeat this experimental study in patient populations in different regions in future studies to further demonstrate the conclusions of this study.

In summary, conventional management combined with case-based nursing management can effectively improve the self-management ability and psychological flexibility of AIDS patients, improve patient care ability and self-efficacy, and provide certain reference value for effective management of AIDS patients.

## Figures and Tables

**Figure 1:** Screening process for included patients.

**Table 1:** Comparison of self-efficacy between the two groups ($\bar{x}\pm s$).

Group	Physical function score		Pain management score		Symptom response score	
	Before intervention	After the intervention	Before intervention	After the intervention	Before intervention	After the intervention
Control group (60)	14.34 ± 3.25	24.25 ± 6.82	8.23 ± 2.57	10.79 ± 3.14	9.16 ± 2.15	19.45 ± 5.15
Observation group (60)	14.73 ± 2.21	33.27 ± 8.31	7.94 ± 1.53	15.23 ± 4.26	8.95 ± 2.26	25.03 ± 8.16
*t*	0.769	-6.499	0.751	-6.499	0.521	-4.479
*P*	0.444	0.000	0.454	0.000	0.603	0.000

**Table 2:** Comparison of the self-management ability of the two groups of patients ($\bar{x}\pm s$).

Group	Symptom management		Emotional cognitive management		Social support and help	
	Before intervention	After the intervention	Before intervention	After the intervention	Before intervention	After the intervention
Control group (60)	28.30 ± 6.23	33.77 ± 4.74	19.23 ± 4.57	22.07 ± 6.14	22.06 ± 3.15	20.45 ± 4.15
Observation group (60)	28.29 ± 5.22	37.37 ± 3.20	19.24 ± 5.53	28.23 ± 4.26	21.95 ± 2.26	28.03 ± 2.16
*t*	0.010	-4.876	-0.011	-6.385	0.220	-12.550
*P*	0.992	0.000	0.991	0.000	0.826	0.000

Group	Daily life management		Disease knowledge management		Treatment compliance management	
	Before intervention	After the intervention	Before intervention	After the intervention	Before intervention	After the intervention
Control group (60)	24.30 ± 6.23	26.29 ± 4.73	12.25 ± 2.53	15.17 ± 2.28	26.41 ± 4.37	30.45 ± 7.19
Observation group (60)	24.29 ± 4.22	30.32 ± 7.27	12.21 ± 1.57	17.60 ± 3.29	26.64 ± 5.27	34.03 ± 3.21
*t*	0.010	-3.599	0.104	-4.702	-0.260	-3.522
*P*	0.992	0.000	0.917	0.000	0.795	0.001

**Table 3:** Comparison of nursing ability scores between the two groups ($\bar{x}\pm s$).

Group	Health knowledge level		Self-care skills		Sense of responsibility	
	Before intervention	After the intervention	Before intervention	After the intervention	Before intervention	After the intervention
Control group (60)	66.40 ± 2.26	65.27 ± 2.14	22.64 ± 6.25	24.25 ± 7.82	12.61 ± 2.51	16.06 ± 2.24
Observation group (60)	66.45 ± 2.22	68.67 ± 4.20	22.66 ± 6.24	61.27 ± 7.61	12.60 ± 2.52	26.65 ± 1.26
*t*	-0.251	-10.689	0.018	-10.669	0.044	-45.064
*P*	0.802	0.000	0.986	0.000	0.965	0.000

**Table 4:** Comparison of nursing ability and mental flexibility between the two groups of patients ($\bar{x}\pm s$).

Group	Toughness		Strength		Optimism	
	Before intervention	After the intervention	Before intervention	After the intervention	Before intervention	After the intervention
Control group (60)	28.40 ± 2.18	31.27 ± 6.29	10.64 ± 2.21	12.25 ± 3.65	7.61 ± 1.48	11.06 ± 2.21
Observation group (60)	28.45 ± 1.27	40.67 ± 5.65	10.66 ± 2.28	24.27 ± 6.66	7.60 ± 1.89	12.95 ± 3.19
*t*	-0.154	-8.612	-0.049	-12.260	0.032	-3.722
*P*	0.878	0.000	0.961	0.000	0.947	0.000

## Data Availability

No data were used to support this study.
